The article "Correlation of Pollen Concentration and Meteorological Factors with Medical Condition of Allergic Rhinitis in Shenyang Area" was published in 2022. Journal: Comput Math Methods Med.

# Correlation of Pollen Concentration and Meteorological Factors with Medical Condition of Allergic Rhinitis in Shenyang Area

**DOI:** 10.1155/2022/4619693

**Published:** 2022-09-27

**Authors:** Feifei Jiang, Aihui Yan

**Affiliations:** Department of Otorhinolaryngology, The First Hospital of China Medical University, Shenyang, 110001 Liaoning, China

## Abstract

**Background:**

The pathogenesis of allergic rhinitis (AR) was affected by meteorological and environmental factors. This study investigated the association between clinical symptoms of AR patients with pollen dispersal and meteorological conditions.

**Methods:**

The clinical features of 10,838 AR patients who were treated in the Department of Otorhinolaryngology, The First Hospital of China Medical University, Shenyang, from March 2021 to October 2021 were retrospectively analyzed. We collected pollen by a pollen collector, read and counted it under a microscope, identified the species of the pollen particles, and recorded meteorological data (average daily temperature, maximum and minimum temperature, average daily wind, average daily precipitation, average daily humidity, average pressure, air quality index, PM2.5, PM10, SO_2_, NO_2_, CO, and O_3_), to analyze the correlation among meteorological conditions, pollen dispersal, and number of AR visits. Finally, pollen allergen-positive and symptoms were scored.

**Results:**

Among the AR visits, patients >41 years old accounted for the highest proportion (64.15%). 43.67% of the patients were complicated with bronchial asthma, and the disease incidence peaked in September. During the period of the study, a total of 27,512 pollen grains were collected, and 17 species were identified. The pollens of Compositae and Moraceae were the main allergenic sources leading to the increase in AR visits from August to September. The peak of pollen dispersal was in spring, summer, and autumn. The total amount of pollen was not only related to the average daily minimum temperature, average daily precipitation, and average daily humidity but also had a significant correlation with air quality index and air pollutants (PM2.5 and PM10, SO_2_, NO_2_, and CO). In addition, there was a significant correlation between the number of daily pollen allergen-positive patients and the pollen concentration of Compositae and Moraceae as well as air pollution components. The clinical symptoms of pollen allergen-positive patients were mainly nasal congestion, red/itchy eyes, and epiphora.

**Conclusion:**

The peak seasons of pollen dispersal in Shenyang were in spring, summer, and autumn, and the allergenic pollens were mainly Compositae and Moraceae. In addition, AR was substantially correlated with pollen concentration and meteorological factors. This study may help provide early warning information and prevention for AR patients.

## 1. Introduction

Allergic rhinitis (AR) is a chronic inflammatory disease of the nasal mucosa caused by reactions in subjects sensitized to allergens mediated by immunoglobulin E (IgE) [1]. AR is also recognized as a global health issue. Recently, the prevalence and incidence of AR have been increasing worldwide, especially in developing countries [2, 3]. AR is commonly classified into seasonal AR (SAR) and perennial AR (PAR), depending on the presence or absence of seasonality and the source of allergens causing its symptoms. SAR has a high incidence in the general population and is an important disease affecting the health of the population. Common clinical features of AR include massive runny nose, sneezing, itchy and congested nose, and occasional itching of the conjunctiva, ears, and throat [4]. Although the symptoms of AR are not life-threatening, they are often disturbing, which affect the quality of work and life and place a heavy burden on individual health and social economy [5, 6]. In addition, it is worth noting that AR often coexists with other allergic diseases, such as asthma and atopic dermatitis [7, 8]. Epidemiological studies have shown that most patients with asthma are associated with rhinitis, and the presence of rhinitis increases the risk factors for asthma [9]. Recently, the number of AR patients in China has increased year by year due to environmental improvement and greening restoration. Therefore, in-depth research is needed to evaluate the epidemiological characteristics and risk factors of AR.

Complex interactions among genes, epigenetics, environmental factors, and lifestyle lead to the occurrence and progression of AR [10, 11]. Airborne allergens such as dust mites, pollen, fungi, and animal dander are widely studied environmental factors affecting allergic reactions [12]. At present, a significant number of studies has reported the risk factors of AR in different regions of the world. For example, Takahashi et al. [13] found that high levels of stress, asthma, atopic dermatitis, tuberculosis, depression, and thyroid disease all increased the risk of AR in the Korean population. In China, An et al. [14] reported that family history of AR, current place of residence, place of residence in infancy, smoking, home decoration, and pet ownership are important risk factors associated with AR prevalence in the general population of Guangzhou. Yang et al. [15] found that self-reported AR prevalence is associated with sinusitis and asthma in the Kazakh population of Fukang, Xinjiang, China, and was mainly positively correlated with carpet use as well as meat and fruit consumption. In addition, air pollutants such as O_3_, NO_2_, and PM are also closely related to the development and deterioration of asthma and AR [12, 16]. For example, high PM10 and PM2.5 concentration aggravates the subjective symptoms of AR in children in Shanghai [17]. It can be seen from the above studies that the causes of AR are various, and it is of great importance to study the etiology of AR for the formulation of effective intervention measures. The purpose of this study was to analyze the risk factors influencing the incidence of AR in Shenyang area and to explore the correlation of pollen concentration and meteorological conditions with the number of AR patients, so as to provide theoretical basis for clinical prevention and treatment of AR.

## 2. Materials and Methods

### 2.1. Subjects

According to the diagnostic criteria, a total of 10,838 AR patients who visited the otolaryngology department of The First Hospital of China Medical University (hereinafter referred to as “our hospital”) from March 1, 2021 to October 18, 2021 were retrospectively analyzed, and the clinical data of the patients were collected from the Electronic Information Center of Hospital. Clinical data of the patients were collected. The inclusion criteria are as follows: patients living in Shenyang for a long time and were diagnosed with AR and patients with no skin scratches, nasal polyps, and chronic sinusitis. The exclusion criteria are as follows: patients with severe eczema and skin abrasions, patients with a history of antihistamine use 20 days prior to enrollment, and patients complicated with mental disorders or autoimmune defects [18]. This study was approved by the Review Committee of our hospital, and the written informed consent was obtained from all participants.

The diagnosis of AR conformed to the clinical diagnosis basis of the “Chinese Guideline for Diagnosis and Treatment of Allergic Rhinitis (2022, Revision)” [19] formulated by the Subspecialty Group of Rhinology, Society of Otorhinolaryngology Head and Neck Surgery, Chinese Medical Association which are as follows:

1. Two or more symptoms of paroxysmal sneezing, clear water-like nasal discharge, nasal itching, and nasal congestion, which persist or accumulate for more than 1 h
2. The nasal mucosa is pale and edematous, and the nasal cavity secretes watery secretions
3. Skin prick test (SPT) detects at least one allergen and/or serum specific IgE-positive, or nasal challenge test-positive

### 2.2. Meteorological and Pollen Data

Meteorological data was daily maximum and minimum temperatures, wind scale, air quality index, PM2.5, PM10, etc. All data are recorded daily by Shenyang Meteorological Station and reported by Shenyang Meteorological Bureau. The pollen data were collected by the pollen monitoring station near the meteorological monitoring station. The pollen collection condition was kept consistent with the climate condition as far as possible. The pollen station was managed by Department of Otorhinolaryngology, The First Hospital of China Medical University. Pollen grains were collected daily using a Durham sampler, which is commonly used in China and counted on a slide under a microscope. Average daily pollen count was used for analysis [20]. Pollen grains were identified based on the *Color Atlas of Airborne Pollen and Plant in China*, the *Pollen Morphology of Tropical and Subtropical Angiosperms in China* (Pollen Morphology Office of South China Institute of Botany), and the *Pollen Morphology of Plants in China* (second edition) [21].

### 2.3. Serum Allergen-Specific IgE (SIgE)

The ImmunoCAP system (Thermo Fisher Scientific, USA) were adopted for serum allergen-specific IgE (SIgE) for all patients. The antigens included dust mites, animal fur, mold, willow, elm, cypress, Oleaceae, walnut, birch, pine, mulberry, ragweed, mugwort, etc. 5 ml of venous blood was first taken from all patients, and the content of serum SIgE was detected with CAP System RAST FEIA enzyme immunofluorescence detector. According to the WHO 75/502 standard, the measurement range was 0.35~100 ku/L, and the CAP test results were divided into 0-6 grades, of which grade 0 was < 0.35 ku/L, level 1 was ≥ 0.35 to < 0.70 ku/L, level 2 was ≥ 0.7 to < 3.5 ku/L, level 3 was ≥ 3.5 to < 17.5 ku/L, level 4 was ≥ 17.5 to < 50.0 ku/L, level 5 was ≥ 50.0 to < 100 ku/L, and level 6 was ≥ 100 ku/L. It was judged as positive by level 1 (≥ 0.35 ku/L) or above.

Subjective clinical symptoms (nasal itching, sneezing, rhinorrhea, nasal congestion, eye redness/itching, and epiphora) were scored for AR patients as follows: nasal itching was 0 for no symptoms, 1 for intermittent nasal itching, 2 for tolerable creeper sensation, and 3 for unbearable creeper sensation; sneezing was 0 for the number of sneezes in one consecutive time < 3, 1 for 3~5 sneezes, 2 for 6~10 sneezes, and 3 for ≥ 11 sneezes. Rhinorrhea was 0 for no symptoms, 1 for ≤ 4 times, 2 for 5~9 times, and 3 for ≥ 10 times (number of nasal blows per day); nasal congestion was 0 for no symptoms, 1 for conscious inhalation, 2 for intermittent or interactive congestion, and 3 for breathing through mouth almost all day; eye redness/itching was 0 for no symptoms, 1 for intermittent eye redness/itching, 2 for obvious but tolerable eye redness/itching, and 3 for persistent and unbearable eye redness/itching; and epiphora was 0 for no epiphora, 1 for a sense of tear filling in the conjunctiva sac but no tear overflow at the eyelid margin, 2 for occasional tear overflow at the eyelid margin, and 3 for frequent or almost continuous tear overflow at the eyelid margin accompanied by nose blowing.

### 2.4. Statistical Analysis

GraphPad software and Excel statistical software were used for all statistical analysis. Counting data were subjected to Pearson correlation analysis to examine the correlation between AR and potential risk factors, and to evaluate the correlation between the daily case number of pollen allergen-positive patients and pollen concentration and air pollutants. *P* < 0.05 was considered to be statistically significant.

## 3. Results

### 3.1. Epidemiological Characteristics of AR

From March 1, 2021 to October 18, 2021, a total of 10,838 AR patients were collected (Table 1). The average age of patients in the cohort was 42 years old (range: 1–99 years old). Among them, 1,734 patients (16.00%) were younger than 18 years old, 2,151 patients (19.85%) were between 18 and 40 years old, 3,489 patients (32.19%) were between 41 and 60 years old, and the remaining 3,464 patients (31.96%) were older than 60 years old. The number of visits was 5,080 (46.87%) for males and 5,758 (53.13%) for females. In addition, 47.91% of patients smoked or had a smoking history, 68.53% of patients kept pets at home, 73.11% of patients grew flowers indoors, and 55.21% of patients had a family history of AR. The number of AR patients complicated with bronchial asthma was 4,733 (43.67%). Meanwhile, the monthly number of cases was counted, and it was found that September had the most visits (20.09%), followed by April (15.62%), March (14.16%), July (14.13%), August (12.16%), May (7.79%), and October (5.53%). The minimum number of visits in October may be related to the fact that the number of visits was only counted up to the 18th day of the month. On the whole, minors accounted for the least proportion of all AR visits, and the proportion of female visits was slightly higher than that of male visits, and nearly half of AR patients had bronchial asthma.

### 3.2. Correlation between Pollen Dispersal and AR

During the study period, a total of 230 films were exposed and 27,512 pollen grains were collected, with an average of 3,439 pollen grains per month. There were three peaks of airborne pollens from March to October, which were from March to April, May, and from August to September. A total of 21,478 pollen grains were collected in spring (March–May), and 6,034 pollen grains in summer and autumn (June–October). The pollen peak period in spring was late March and mid-May, and the pollen peak period in summer and autumn was August (Figure 1(a)). The known pollen species recorded in the exposed film included 17 species, which were Salicaceae, Ulmaceae, Gramineae, Cupressaceae, Ginkgoaceae, Oleaceae, Juglandaceae, Betulaceae, Pinaceae, Leguminosae, Moraceae, Rosaceae, Urticaceae, Cyperaceae, Compositae, Amaranthaceae, and Chenopodiaceae. The fragmented and unidentifiable pollens were classified as others. Among the 17 pollen species, 9 types of dominant pollens were found, among which the dominant pollens in spring were Salicaceae, Pinaceae, Ulmaceae, Cupressaceae, Rosaceae, Oleaceae, and Ginkgoaceae, and the dominant pollens in summer and autumn were Compositae and Moraceae (Figure 1(b)). Then, the pollen concentration and outpatient visits of AR patients from March to October 2021 were analyzed. It was found that the trend of the number change of AR visits and the trend of pollen concentration change were inconsistent in time, and the number of cases was obviously divided into three periods: from March to mid-May, from June to July, and from September to October. However, we found that the number of visits of AR patients in summer and autumn was significantly higher than that in spring, and the number of cases peaked in September (Figure 1(c)). Due to the significant differences in pollen dispersal in different seasons found above, we conjectured that AR prevalence might be associated with pollen species. Combined with the analysis of pollen species distribution characteristics, it was found that although the pollen concentration of Salicaceae accounted for the highest proportion of all pollens (40.85%), the number of visits of AR patients was not high in the peak period of dissemination of Salicaceae. However, with the increase of pollen concentration of Compositae and Moraceae, the number of visits to AR patients increased significantly in summer and autumn. Subsequently, we conducted correlation analysis on the daily total pollen concentration of Compositae, Moraceae, and Salicaceae and AR outpatient visits (Table 2). We found that both the daily total pollen concentration and Salicaceae pollen concentration had no correlation with AR outpatient visits (*P* > 0.05), while Compositae and Moraceae pollen concentration had a positive correlation with AR outpatient visits (*P* < 0.05, Table 2). Based on the above analysis, Compositae and Moraceae were the main allergenic herbaceous pollens for AR in summer and autumn.

### 3.3. Relationship of Meteorological Conditions and Pollen Dispersal with AR

In addition to the internal factors such as the condition of regional vegetation, the law of plant growth and development, and the characteristics of pollen itself, the external meteorological factors also affect the law of airborne pollen dispersal. Meteorological elements (including daily average temperature, daily average minimum or maximum temperature, daily average wind, daily average precipitation, daily average relative humidity, and daily average atmospheric pressure) and air pollution status (including air quality index, PM2.5, PM10, SO_2_, NO_2_, CO, and O_3_) in Shenyang from March 2021 to October 2021 as well as total pollen count and number of AR patients in the same period were enrolled for statistical analysis (Table 3). It could be seen that total pollen count was significantly correlated with daily minimum temperature, average daily precipitation, and average daily relative humidity (*P* < 0.05), but not with daily average temperature, maximum temperature, average atmospheric pressure, and wind scale (*P* > 0.05). In addition, total pollen count had a significant correlation with air quality index, PM2.5, PM10, SO_2_, NO_2_, and CO (*P* < 0.05), indicating that pollen dispersal was one of the factors contributing to the increase of the concentration of these adverse pollutants in the air. It was worth noting that there was no correlation between the number of AR cases and meteorological factors (*P* > 0.05). Therefore, we concluded that the change of meteorological conditions was one of the factors that make pollen become the main allergen of AR.

### 3.4. Correlation of the Number of Daily Pollen Allergen-Positive Patients with Air Pollution Components and Pollen Concentration

A total of 7,931 (73.18%) positive patients were detected from March 1, 2021, to October 18, 2021, including 4,364 males (55.02%) and 3,567 females (44.98%). The number of positive cases per month from March to October were 349, 582, 737, 534, 639, 3418, 1449, and 223, respectively. We conducted statistical analysis on the daily total pollen concentration, pollen concentration of Compositae, Moraceae, and Salicaceae, and the daily number of pollen allergen-positive patients, and the results were shown in Figure 2. The yellow line presents the number of allergen-positive patients per month, which was consistent with the curve of pollen concentration of Compositae and Moraceae but significantly different from the curve trend of total pollen concentration and pollen concentration of Salicaceae. This further confirmed that Compositae and Moraceae were the main allergenic pollen of AR in Shenyang area. In addition, there was a weak correlation between the daily number of pollen allergen-positive patients and the total daily pollen concentration (*P* = 0.043), while the daily case number was significantly correlated with the pollen concentration of Compositae and Moraceae (*P* < 0.001) but not with the pollen concentration of Salicaceae (Table 4). Meanwhile, correlation analysis was conducted between the concentration of 6 kinds of air pollutants and the daily number of pollen allergen-positive patients, and significant correlations were found between the daily number of patients and the daily concentration of pollutants PM2.5, PM10, SO_2_, and NO_2_(*P* < 0.05) (Table 4).

### 3.5. Pollen Allergen-Positive and Symptom Score

According to the results of pollen allergen test, AR patients were divided into the positive group and the negative group, and the clinical symptoms of the two groups were compared. The results were shown in Table 5. There were statistically significant differences between the positive group and the negative group in nasal congestion, eye red ness/itching, and epiphora symptom scores (*P* < 0.05), while no significant differences were seen in nasal itching, sneezing, and rhinorrhea between the two groups (*P* > 0.05). Additionally, the three symptoms of nasal congestion, eye redness/itching, and epiphora were more pronounced in the pollen allergen-positive group than in the negative group.

## 4. Discussion

In the past decade, the incidence of AR in China has been on the rise, especially in densely populated cities [22]. However, the reasons for the rapid increase of the incidence of AR are not completely clear at present, and it is urgent to find the reasons for AR increase and make appropriate countermeasures. Although there have been several epidemiological studies on AR in major cities in China, the allergen characteristics of AR patients in different regions and ages in China differ greatly due to the vast territory and large population [23, 24]. Improved sanitation, increased allergen exposure, and changes in dietary habits and lifestyle may increase the prevalence of AR [13, 25]. Therefore, it is of great importance for the prevention and treatment of AR to understand the distribution characteristics of allergens and related risk factors in each region. The present study analyzed the factors influencing the number of AR outpatient visits among the general population in Shenyang, China from March 1 to October 18, 2021. Our study showed that the AR consultation rate of middle-aged people aged 41–60 in Shenyang was the highest, and the gender difference was not significant, but the female rate was slightly higher than the male rate. Similarly, Hong et al. [26] analyzed the prevalence of AR in Guangzhou and Zhuhai in Southern China, and they found that there was no significant gender difference, but the incidence of AR in males was slightly higher than that in females. Therefore, we guessed that gender was not the primary risk factor for AR. In addition, it is worth noting that nearly half of the AR patients in the present study were complicated with bronchial asthma. This is consistent with the results reported in previous studies that asthma and AR are usually comorbidities and coexist in the same patient in China [27]. Previous studies have shown that AR is an independent risk factor for the development of asthma or other dangerous respiratory diseases in individuals [28]. Therefore, knowing more about the risk factors associated with AR can help improve symptoms and quality of life and reduce asthma exacerbation in patients with coexisting asthma and persistent AR.

Pollen has been reported to be an important cause of seasonal AR, and typical pollens involved include wind-pollinated trees and grasses [29]. Recently, with the improvement of the environment, pollen concentration has been increasing year by year in major cities in China, and pollen-related allergens have attracted the attention of many scholars in China. A study investigated the prevalence of AR caused by high pollen exposure in the grasslands of northern China and found that the incidence of AR caused by pollen was very high in the investigated area due to the influence of local environmental and climatic conditions [30]. Zhang et al. [31] found that with the increase of pollen concentration in ambient air, the relative risks on daily number of outpatients of AR were increased. Thus, high pollen level was a risk factor for the development of AR symptoms. However, there was no report on the effect of airborne pollen on AR visit frequency of Shenyang residents. In this study, it was found that there were two obvious peak periods of pollen distribution in Shenyang area, one in spring (from March to May) and the other in summer and autumn (from June to October). The actual temperature in these two periods could increase the yield and concentration of pollen and enhance the antigenicity of pollen [17, 32]. Interestingly, in this study, there was no linear correlation between the daily total pollen concentration and the daily number of AR patients, and the number of AR patients in spring was significantly lower than that in summer and autumn, which may be due to the fact that the dominant Salicaceae pollen disseminated in spring is not an important source of allergens [33]. On the contrary, the number of AR visits peaked in August and September. During the same period, the pollen concentration of Compositae and Moraceae increased significantly. This is consistent with the results of Bishan et al. [21] that Moraceae, Artemisia in Compositae, and Gramineae are the main allergenic pollen types, with peak concentrations from April to May, from August to September, and from October to December, respectively [21]. Additionally, the positive result of pollen SIgE showed that the number of pollen-allergen positive AR patients during pollen seeding period was significantly positively correlated with the concentration of Compositae and Moraceae pollen in the air, which might be because AR patients allergic to these two kinds of pollen had higher sensitivity to SIgE during pollen seeding period. Therefore, we believed that Compositae and Moraceae were the most important herbaceous plants with allergenic pollen in Shenyang area. It has been reported that pollen allergy is significantly related to the symptom severity of rhinitis patients [34]. By analyzing the clinical symptoms and characteristics of AR patients, it was found that patients with positive pollen allergen had more evident symptoms of nasal congestion, eye redness/itching, and epiphora. It is easy to cause allergic reactions in the mucous membrane when pollen falls down into the eyes or is inhaled through the nose and pharynx. Therefore, patients with positive pollen allergen had more obvious accompanying ocular symptoms and nasal congestion than those in negative patients. The subsequent study will further perfect the symptoms and objective evaluation indicators, and the related causes and pathogenesis will be analyzed.

Since the nature and quantity of pollen varies with vegetation, geography, temperature, and climate, the sensitivity of people in different areas to pollen species is different [35]. Studies have shown that changes in weather conditions such as rainfall, atmospheric temperature, humidity, wind speed, and wind direction can change the seasonality and concentration of plant pollen, thus inducing allergic symptoms and leading to the occurrence and development of AR [36–38]. Temperature plays a very important role in increasing the pollen concentration in the air and is the main factor controlling the start of grass pollen season and the peak duration of pollen [21, 39, 40]. In the present study, we found that total pollen amount in Shenyang significantly correlated with daily minimum temperature, daily average precipitation, and daily average relative humidity but not with daily average temperature, maximum temperature, average atmospheric pressure, and wind scale. In fact, it is difficult to explain the correlation between pollen concentration and meteorological parameters, because the relationship between pollen and meteorological conditions can be nonlinear. Pollen concentration can be affected by multiple meteorological conditions at the same time, so it is difficult to make correlation tests. We assumed that the meteorological conditions shown in the present paper were not correlated with pollen concentration based on the above reasons [21, 41]. In addition, the concentration of air pollutants (such as SO_2_, NO_2_, CO, and O_3_) was consistent and significantly correlated with the concentration of grass pollen in the air [42]. In this study, the results show that total pollen amount had a significant correlation with the concentrations of PM2.5, PM10, SO_2_, and NO_2_ in Shenyang area, which is also confirmed at this point. Moreover, there were also significant correlations between the number of pollen allergen-positive patients and the daily concentrations of PM2.5, PM10, SO_2_, and NO_2_. Based on the above studies, it can be concluded that allergenic pollen could mediate AR consultation rate through local meteorological conditions.

In summary, this study illustrated how pollen dispersal, climate change, and outdoor air pollution acted as the environmental risk factors for AR development in Shenyang area. To be specific, the lower temperature from August to September was conducive to the pollen dispersal of Compositae and Moraceae, leading to the increase of particulate pollutants in the air and the deterioration of air quality, which leads to a significant increase in outpatient visits of AR patients in the same period. This study had a large sample size, which could reflect the whole AR consultation laws and the relevant air environmental factors in Shenyang area. However, clinical data collection of subjects in the cohort was incomplete, and the impact of other risk factors, such as residential habits and occupational dust exposure and allergy history, on AR is still unclear. Subsequently, clinical data of patients should be improved to comprehensively analyze multiple factors affecting AR consultation rate, providing reference materials for clinical prevention and treatment of AR.

## Figures and Tables

**Figure 1:** Correlation between pollen dispersal and AR. (a) Variation trend of airborne pollen concentration during pollen dispersal period. (b) Distribution of dispersal of dominant pollens. (c) Number of visits for AR and trend of pollen concentration variation.

**Figure 2:** Correlation between the number of pollen allergen-positive patients per month and pollen concentration.

**Table 1:** Clinical features of AR in Shenyang area.

Characteristics	Number (n)	Percentage (%)
Age (years)		
<18	1734	16.00
18–40	2151	19.85
41–60	3489	32.19
>60	3464	31.96
Gender		
Male	5080	46.87
Female	5758	53.13
Smoking habit		
Never smoking	5645	52.08
Now smoking	3550	32.75
Ever smoking	1643	15.16
Keeping pets		
Yes	7427	68.53
No	3411	31.47
Family history of AR		
Yes	5983	55.21
No	4855	44.79
Indoor flower cultivation		
Yes	7923	73.11
No	2915	26.89
Combined diseases		
Bronchial asthma	4733	43.67
Nonbronchial asthma	6105	56.33
Month		
March	1535	14.16
April	1693	15.62
May	844	7.79
June	1140	10.52
July	1531	14.13
August	1318	12.16
September	2177	20.09
October	600	5.53

**Table 2:** Correlation analysis of pollen dispersal and allergic rhinitis.

Pollen concentration	Number of patients	
	R^2^	*P* value
Total concentration	0.01388	0.0733
Compositae	0.05165	0.0005
Moraceae	0.1029	<0.0001
Salicaceae	0.003098	0.3987

**Table 3:** Correlation analysis of meteorological conditions with pollen dispersal and allergic rhinitis.

Meteorological elements	Pollen concentration		Number of patients	
	R^2^	*P* value	R^2^	*P* value
Average temperature	0.01087	0.1133	0.001782	0.5223
Minimum temperature	0.01789	0.0418	3.605e-005	0.9275
Maximum temperature	0.004501	0.3089	0.006541	0.2197
Average wind	0.007776	0.1807	0.0001071	0.8754
Average daily precipitation	0.244036	<0.0001	0.01344	0.09
Average daily humidity	0.106276	<0.0001	0.014641	0.066
Average pressure	0.000676	0.695	0.013689	0.075
Air quality	0.06817	<0.0001	0.0008591	0.6570
PM 2.5	0.05973	0.0002	0.0006355	0.7025
PM 10	0.1211	<0.0001	0.002178	0.4793
SO_2_	0.1654	<0.0001	0.008125	0.1712
NO_2_	0.08412	<0.0001	0.01568	0.0569
CO	0.05527	0.0003	0.005179	0.2750
O_3_	0.01140	0.1048	0.003550	0.3663

**Table 4:** Correlation of the number of daily pollen allergen-positive patients with air pollution components and pollen concentration.

Elements	Number of daily pollen allergen-positive patients	
	^R^2	*P* value
Total concentration	0.017689	0.043^∗^ (<0.05)
Compositae	0.429025	<0.001
Moraceae	0.370811	<0.001
Salicaceae	0	0.994
PM2.5	0.0441	0.001^∗^ (<0.05)
PM10	0.057121	<0.001
^SO^_2_	0.26244	0.014^∗^ (<0.05)
^NO^_2_	0.016641	0.04^∗^ (<0.05)
CO	0.014641	0.066
^O^_3_	0.007225	0.199

∗Represents *P* < 0.05.

**Table 5:** Pollen allergen-positive grouping and symptom score.

Symptom	Pollen allergen-positive	Pollen allergen-negative
Nasal itching	1.86 ± 0.95	1.69 ± 1.03
Sneezing	2.32 ± 0.93	2.14 ± 0.93
Rhinorrhea	2.15 ± 1.01	1.97 ± 0.97
Nasal obstruction	2.24 ± 0.89	1.9 ± 0.92^a^
Red eye/itching	1.98 ± 0.94	1.23 ± 0.89^a^
Epiphora	1.36 ± 0.97	0.86 ± 0.91^a^

Compared with the pollen allergen-positive group, ^a^ represents *P* < 0.05.

## Data Availability

All data generated or analyzed during this study are included in this article.
